The article "Study on the Influence of Compression Ratio on the Rail Contact Fatigue Resistance Property and Its Mechanism" was retracted in 2023. Reasons: signs of a paper mill; compromised peer review; unreliable results or conclusions.

# Study on the Influence of Compression Ratio on the Rail Contact Fatigue Resistance Property and Its Mechanism

**DOI:** 10.1155/2021/9057677

**Published:** 2021-10-29

**Authors:** Zhiqiang Li

**Affiliations:** ^1^College of Materials Science and Engineering, Chongqing University Chongqing, 400030, Chongqing, China; ^2^Pangang Group Research Institute Co., Ltd., Panzhihua 617000, Sichuan, China

## Abstract

Contact fatigue resistance properties of four commercial steel rails were systematically studied and compared. The contact fatigue limit cycles, fracture toughness, and fatigue crack growth rate of the corresponding rails with different compression ratios were tested and analyzed, which showed a close relationship between them. Moreover, microstructures of the rails were carefully observed by using the TEM to elucidate the scientific mechanisms. Observations and obtained results indicated that pearlite lamellar spacing further decreased with the rise of compression ratio, which greatly and rightly contributed to the improved fatigue resistance property.

## 1. Introduction 

Rolling contact fatigue is an inevitable phenomenon in the process of wheel-rail service. Contact fatigue is one of the main failure modes of rails [1]. With the improvement of contact conditions, the surface wear trend of the wheel-rail system decreases gradually, while the contact fatigue damage of the subsurface becomes more and more serious [2]. In the process of wheel-rail contact, for rails, the shear plastic deformation can be as high as 100%, and the depth of the deformation layer can reach about 2 mm [3]. As a result of plastic deformation, cavities or microcracks are initiated at subsurface defects. With the continuous accumulation of plastic deformation, adjacent cavities aggregate with each other, and microcracks grow up, thus forming macroscopic cracks [4]. In order to explore the relationship between the rail contact fatigue resistance property and rail compression ratio, this paper conducts a systematic study on the rail contact fatigue resistance property of four different compression ratios. By systematically observing the microscopic internal organization of rails, the mechanism of the influence of rail compression ratio on its contact fatigue resistance property is analyzed.

## 2. Test Materials and Methods

### 2.1. Test Materials

The test material is a heat-treated rail produced by a domestic steel plant, the grade is U78CrV, and its chemical composition is shown in Table 1.

### 2.2. Test Method

The U78CrV heat treatment rails with compression ratios of 11.1, 13.6, 13.8, and 17.1 were tested for fatigue resistance property indicators such as contact fatigue limit cycles, fracture toughness, and fatigue crack growth rate.

#### 2.2.1. Contact Fatigue Limit Cycle Test

The test sample is taken at the head of the rail, and the physical contact fatigue test is carried out using the two-wheel-to-roll method using Ansys simulation to calculate the test contact stress, as shown in Figure 1.

When the test speed is 750 rpm, the sample can be damaged in a short time. At the same time, the angular speed of 750 rpm corresponds to the speed of about 120 km/h of the train with 840 mm diameter wheels, which is closer to the real situation. In order to get as close as possible to the slip condition of the line, a minimum 5% slip is used to carry out the test. Taking all factors into consideration, the laboratory conducts contact fatigue tests. The parameters are shown in Table 2.

#### 2.2.2. Fracture Toughness Test

Take rail fracture toughness samples at the rail head positions corresponding to each compression ratio. The sampling positions are shown in Figure 2. The sample width *W* is 40 mm, the sample length is 180 mm, and the letter “H” is printed on the end of the sample.

After the sample processing is completed, the sample is subjected to wire cutting to process the overall knife edge and precrack. The testing equipment used is the INSTRON 8801 electrohydraulic servo material testing machine. The test temperature is −20°C.

#### 2.2.3. Fatigue Crack Growth Rate Test

The fatigue crack growth rate sampling of rails corresponding to different compression ratios is carried out at the position of the rail head. The sampling positions and processing dimensions of the samples are shown in Figures 3 and 4.

The processed fatigue crack growth rate samples are tested. The inspection equipment is an INSTRON 8801 fully digital-controlled electrohydraulic servo material testing machine. The inspection temperature is −20°C. During inspection, span *S* = 4°W, load ratio *R* = 0.5, sinusoidal waveform, and load frequency *f* = 30 Hz.

## 3. Test Results

### 3.1. The Influence of Compression Ratio on Rail Contact Fatigue Limit Cycles

Figure 5 shows the sound decibel recording curve during the contact fatigue test. It can be seen from the figure that the whole test process can be divided into A and B sections. At the initial stage of the test, in section A, the sound decibel was relatively stable. This indicates that the surface of the sample is relatively smooth and flat at this stage. As the number of cycles increases, microcracks and other changes appear on the surface of the sample, which make the test decibel increase slightly. In section B, when the surface of the sample is peeled off, the sound decibel increases rapidly. This indicates that the sample is damaged at this stage, and as the cycle times increase, the damage becomes more serious, and the test decibel increases rapidly. The intersection of two segments A and B is the critical point at which fatigue failure occurs, that is, the fatigue limit cycle.

Under different contact stress conditions, the rail fatigue limit cycles corresponding to each compression ratio were measured. The results are shown in Table 3, and the change trend is shown in Figure 6.

It can be seen from Table 3 and Figure 6 that the number of cycles of the rail contact fatigue limit increases with the increase of compression ratio. When the contact stress reaches 1628 MPa, the rail contact fatigue cycles show a linear increase in the compression ratio.

### 3.2. The Influence of Compression Ratio on Rail Fracture Toughness

The test results of the fracture toughness of each compression ratio corresponding to the rail are shown in Table 4. Its changing trend is shown in Figure 7.

It can be seen from Table 4 and Figure 7 that the rail fracture toughness generally increases with the increase in compression ratio. Among them, rail compression ratios of 13.6 and 13.8 are close to the rail fracture toughness values.

### 3.3. The Effect of Compression Ratio on Rail Fatigue Crack Growth Rate

The fatigue crack growth rate test results of each compression ratio corresponding to the rail are shown in Table 5. Their changing trends are shown in Figure 8.

It can be seen from Table 4 and Figure 8 that the rail crack growth rate shows a significant downward trend with the increase of compression ratio.

## 4. Mechanism Analysis

The basic process of contact fatigue is as follows: under the action of contact stress, plastic deformation occurs on the surface or subsurface, which leads to damage and contact fatigue crack with the accumulation of damage. According to Smith's theory, the mechanical conditions for the formation of cracks in cementite sheets are [5]

(1) $$\begin{array}{c} \tau_{eff}\geq {\left[\frac{4E\gamma_{c}}{\pi a\left(1-v^{2}\right)}\right]}^{1/2}. \end{array}$$

In the formula, *τ*_eff_ is the critical effective shear stress when cementite cracks.

 
*γ*_*c*_ is the surface energy of cementite
  E is the positive modulus of elasticity of cementite
  v is Poisson's ratio
 
**a** is the ferrite sheet thickness

According to formula (1), it can be seen that the critical effective shear stress, when cementite cracks, is inversely proportional to the square root of the ferrite sheet thickness. Furthermore, it can be approximated that it is inversely proportional to the square root of the pearlite interlayer spacing. Clyton [6] and Kalousek and Laufer [7] also reported similar test results. Based on this theory, the internal structure of the sample before and after the contact fatigue test was observed by using the transmission electron microscope, and the pearlite lamellar spacing before and after the test was measured. The results of the measurement and observation are shown in Table 6 and Figure 9.

It can be seen from Table 6 and Figure 9 that the interlayer spacing of rail pearlite tends to decrease with the increase of compression ratio. The interlayer spacing of pearlite decreased after contact fatigue test. The smaller the rail between the original lamellae, the greater the reduction of the lamellar interval. This shows that its plastic deformation ability is stronger. It can be seen from the deformed structure of the sample after the test that the rail pearlite lamellar spacing with a compression ratio of 11.1 is the largest. Its cementite sheet broke. Rail pearlite sheets with compression ratios of 13.6 and 13.8 have moderate spacing. Their cementite showed bending deformation and a small amount of fracture. The rail pearlite sheet with a compression ratio of 17.1 has the smallest interlayer spacing, and its cementite sheet has been slightly bent and deformed without breaking. It can be seen that the smaller the distance between the original pearlite sheets, the less prone to fracture of its cementite sheets and the higher the contact fatigue resistance property. The greater the distance between the original pearlite sheets is, the more likely it is that the cementite sheets will break, and the contact fatigue resistance property is relatively low.

## 5. Conclusion

1. As the rail compression ratio increases, the contact fatigue limit cycles and fracture toughness of the corresponding rail gradually increase. The crack growth rate of the rail shows a downward trend; that is, the contact fatigue resistance property of the rail is improved.
2. Observed by using the transmission electron microscope, the larger the compression ratio of the rail, the finer the distance between the original pearlite sheets of the rail. After the rail contact fatigue test, the rail pearlite layer spacing corresponding to each compression ratio has been reduced. The cementite in pearlite is deformed and fractured.
3. The larger the distance between the original pearlite sheets of the rail is, the more easily the cementite sheets will be deformed and fractured. Its fatigue resistance property is relatively low. The finer the distance between the original pearlite sheets is, the less the cementite sheet is susceptible to bending deformation and fracture, and it has a relatively high contact fatigue resistance property.

## Figures and Tables

**Figure 1:** Two-wheel-to-roll model of the laboratory.

**Figure 2:** Sampling location of fracture toughness samples.

**Figure 3:** Sample location of fatigue crack growth rate.

**Figure 4:** Processing size of the fatigue crack growth rate specimen.

**Figure 5:** Test sound curve.

**Figure 6:** The trend of rail contact fatigue limit cycles with compression ratio.

**Figure 7:** Trend of rail fracture toughness with compression ratio.

**Figure 8:** Trend of fatigue crack growth rate with compression ratio.

**Figure 9:** Transmission electron microscope observation of the sample before and after the contact fatigue test. (a) Before the test. (b) After the test.

**Table 1:** Chemical composition of test materials (%).

Grade	C	Si	Mn	P	S	Cr	V	Al
U78CrV (R)	0.79	0.72	0.82	0.013	0.006	0.33	0.08	0.004

**Table 2:** Test plan for contact fatigue cycles.

Scheme	Contact stress (MPa)	Rotational speed (rpm)	Slip (%)
One	1377	750	5
Two	1502	750	5
Three	1628	750	5

**Table 3:** Each compression ratio corresponds to rail contact fatigue limit cycles/10,000 times.

Contact stress (MPa)	Contact fatigue limit cycles/10,000 times			
	*R* = 11.1	*R* = 13.6	*R* = 13.8	*R* = 17.1
1377	61.9–69.8	63.8–75.2	64.3–75.5	69.4–79.8
	66.5	69.3	70.1	75.3

1502	56.9–60.5	59.8–67.4	59.6–68.7	62.6–73.1
	58.9	63.5	63.9	67.7

1628	41.2–44.4	42.7–47.3	43.2–48.9	44.8–52.3
	42.6	44.9	46.5	48.4

**Table 4:** Each compression ratio corresponds to rail fracture toughness.

Compression ratio	KIC (MPa m^1/2^)
11.1	30.16–34.33
	32.03

13.6	32.37–36.5
	34.25

13.8	31.72–35.52
	33.22

17.1	32.54–37.85
	35.61

**Table 5:** Corresponding rail fatigue crack growth rate of each compression ratio.

Compression ratio	d*a*/d*n*, mm/cycle (Δ*K* = 10 MPa m^0.5^)	d*a*/d*n*, mm/cycle (Δ*K* = 13.5 MPa m^0.5^)
11.1	(10.9–16.6) × 10^−6^	(32.8–39.3) × 10^−6^
	13.7 × 10^−6^	36.4 × 10^−6^

13.6	(10.4–15.3) × 10^−6^	(31–37.4) × 10^−6^
	12.5 × 10^−6^	34.7 × 10^−6^

13.8	(9.1–12.6) × 10^−6^	(26.2–31.5) × 10^−6^
	10.3 × 10^−6^	28.9 × 10^−6^

17.1	(6.5–10.8) × 10^−6^	(23.7–26.6) × 10^−6^
	8.7 × 10^−6^	25.2 × 10^−6^

**Table 6:** Each compression ratio corresponds to rail pearlite interlayer spacing (nm).

Compression ratio		11.1	13.6	13.8	17.1
Pearlite interlayer spacing (nm)	Before the test	169	143	138	113
	After the test	150	106	97	72
	Reduction rate (%)	11.2	25.9	29.7	34.5

## Data Availability

The data that support the findings of this study are available upon request to the author.
